# SOC Estimation of Lithium-Ion Battery for Electric Vehicle Based on Deep Multilayer Perceptron

**DOI:** 10.1155/2022/3920317

**Published:** 2022-05-16

**Authors:** Xueguang Li, Haizhou Jiang, Sufen Guo, Jingxiu Xu, Meiyan Li, Xiaoyan Liu, Xusong Zhang

**Affiliations:** ^1^China Research Institute of Radiowave Propagation, Xinxiang, Henan Province 453000, China; ^2^School of Fine Arts, Xinxiang University, Xinxiang, Henan Province 453000, China; ^3^School of Computer, Huanggang Normal University, Huangang, Hubei Province, China; ^4^School of Information Engineering, Baise University, Baise, Guangxi Province 533000, China; ^5^Department of Virtual Reality, Jiangxi Tellhow Animation Vocational College, Jiangxi Province 330200, China; ^6^Guizhou Coalfield Geology Bureau, Guiyang, Guizhou Province 550000, China

## Abstract

The state of charge (SOC) is one of the main indexes of the lithium-ion battery, which affects the practice range of new energy vehicles and the safety of the battery. Nevertheless, the value of SOC cannot be measured directly. At present, the algorithm for estimating the state of charge is not very satisfactory. The multilayer perceptron algorithm designed during this paper encompasses a sensible impact on state estimation. During this paper, the multilayer network is designed to estimate the charged state of lithium batteries from the three-layer artificial neural network to the eleven-layer artificial neural network. After preprocessing the dataset and comparing several activation functions, the ten-layer fully connected neural network is the most efficient to estimate the SOC. In order to prevent over-fitting of the multilayer perceptron algorithm, the two techniques of the BatchNormalization layer and Dropout layer work together to inhibit over-fitting. At the same time, the accuracy of extended Kalman filter, long and short memory network, and recurrent neural network are compared. The multilayer perceptron network designed during this paper has the highest accuracy. Finally, in the open dataset, both the training and test errors achieve good results. The algorithm developed in this paper has made some progress in SOC estimation.

## 1. Introduction

Since the twenty-first century, the energy crisis [1], automobile exhaust pollution, and alternative issues became progressively outstanding, and reducing carbon emissions has become an agreement. Environmentally friendly vehicle suggests that transport has so ushered in unprecedented development opportunities. As a “zero-emission” vehicle, new energy vehicles have attracted international attention. In addition, the development of pure electric vehicles [2] is very rapid. The main reason is the energy data storage medium used in electric vehicles–lithium-ion battery [3]. Lithium-ion batteries have the advantages of long cycle life, high energy density, and low internal resistance.

Nevertheless, the lithium-ion battery has typically been concerned in severe accidents, like the explosion of telephones, whereas charging and therefore the spontaneous combustion of automotives. These batteries run the risk of overcharging or over-discharging. These problems can lead to battery overheating and spontaneous combustion, and these problems have received a lot of attention. In order to reduce or eliminate these problems, the battery management system plays a critical role. In the battery management system [4], the accuracy of battery state of charge (SOC) estimation is an important indicator to measure battery performance. SOC is one of the critical parameters of lithium-ion batteries. The more accurate the battery SOC estimation, the better the performance of the battery management system. Accurate SOC estimation can not only reflect the battery's remaining capacity but also effectively prevent battery risks in advance. It can not only ensure the safety of pure electric vehicles but also ensure the safety of human life. Therefore, the research on SOC estimation is of great significance.

## 2. Related Work

The estimation methods of SOC can be divided into three categories [5, 6]. The first category is the simple table lookup method [5, 6], which is mainly represented by the ampere-hour integration method and open-circuit voltage method [7]. These methods are mainly by making a table of the OCV-SOC [8] corresponding curve. The microcontroller can modify and estimate SOC simply by looking up the table. This method is usually used in conjunction with ampere-hour integration. The ampere integral method uses dynamic estimation. The magnitude of the discharge current is integrated according to time. The remaining charge is then calculated by subtracting the initial charge from the integral. The ratio of the remaining power to the initial power is the value of SOC. This simple lookup table method [9] is widely used in engineering. However, the estimation error of this method is large, and it cannot be used for fast real-time estimation. The second category is model-based SOC estimation methods [10]. Due to the internal complexity of the battery, there is no ready-made model for use. This direction is equivalent to the battery by building its model. The SOC estimation in the model is used to replace the SOC estimation of the battery. There are several approaches to this direction. Electrochemical Model (EM) [11] is a battery model based on the porous electrode and solution concentration theory, which are mainly based on the electrochemical reaction process to calculate the terminal voltage and SoC of the battery. In addition, Electrochemical Impedance Model (EIM) [12] was developed. Electrochemical impedance spectroscopy (EIS) [13] is also commonly used as a model for estimating SOC. EIM and EIS both believe that there is a certain correspondence between battery impedance and SOC. The SOC can be accurately estimated by measuring and calculating the battery's impedance.

Equivalent Circuit Model (ECM) [13–15] is used to describe and simulate the dynamic characteristics, which are treated as a two-port network. Standard models include the Rint model, Thevenin model, and Partnership for a New Generation of Vehicle (PNGV) model [15]. The curve fitted by the model-based SOC estimation method has a higher matching degree with the real voltage curve. Still, the circuit model becomes more complex, and the increase of parameters makes parameter identification more challenging to achieve. ECM is simple in structure and easy to calculate. Researchers often combine ECM with adaptive algorithms such as the Kalman filter to estimate battery SOC. The third category is a data-driven estimation. The data-based estimation method refers to the direct estimation of SOC using battery data by measuring battery parameters such as current, voltage, temperature, and internal resistance. With the rapid development of machine learning and deep learning, data-driven SOC estimation methods often use the machine learning platform. Intelligent algorithms automatically learn network parameters and obtain the relationship between electricity pool parameters and SOC. Machine Learning methods commonly used for SOC estimation include neural network and deep learning algorithm, Support Vector Machine (SVM) [7], and Extreme Learning Machine (ELM) [9, 16].

All of those strategies can estimate the SOC of lithium-ion batteries. However, these estimation algorithms become additional and inaccurate with the period of lithium-ion batteries. The main disadvantages of the ampere-hour integration method and the open-circuit voltage method are time-consuming, low efficiency, and low precision. The ampere-hour integration method and the open-circuit voltage method have not been able to form a closed loop. The most disadvantage of the second category of model-based estimation strategies is the issue of modeling. It conjointly has some disadvantages like the severe parameter identification problem and an oversized quantity of calculations. The third category could be a data-driven estimation. Its main disadvantages are the high demand for information and the long training time. Owing to these shortcomings, in this paper, the estimation of lithium-ion batteries uses the algorithm based on a multilayer perceptron. It uses open datasets. It can compute on computers and in cloud servers, making computing very fast because of the excellent performance of cloud servers and computers. In order to meet the optimal estimation of SOC training error and testing error of lithium-ion battery, different multilayer perceptron depth is designed in this paper. The SOC is calculable by the multilayer perceptron algorithm designed during this paper. They can do sensible accuracy. The algorithm designed during this paper will promote the correct estimation of SOC. It has a massive impact on the range and safety of pure electric vehicles. Additionally, the algorithm designed during this paper can also be applied to alternative fields like mining machinery and instrumentation state assessment, metallurgic instrumentation running state assessment, etc.

## 3. Method

### 3.1. The Definition of SOC

In general, SOC [3, 17, and 18] is the ratio of the remaining electric quantity to the rated electric quantity. Lithium-ion batteries have typical nonlinear characteristics, and it is difficult to measure the total power released by existing means or methods. According to the theory of ampere-hour integration, SOC is particularly critical because it can accurately reflect the energy state, and its calculation formula is as follows:

(1) $$\begin{array}{c} \text{SOC}=\frac{Q_{c}}{Q_{0}},\\ \text{SOC}=1-\frac{Q_{T}}{Q_{0}}. \end{array}$$

*Q*_*c*_ is the remaining electric quantity, and *Q*_0_ is the initial electric quantity at a certain temperature or the rated charge at a certain temperature. *Q*_*T*_ is how much electric quantity of the battery has already been released. The definition of the calculation form of the ampere-hour integral method is generally used in the calculation process. There is no direct way to measure the amount of electric quantity released by a lithium-ion battery during a real process. Therefore, under the circumstances, it is based on the discharge current integral accumulative as the release of electric quantity.

(2) $$\begin{array}{c} \text{SOC}\left(t\right)=SOC_{0}-\frac{\int_{0}^{t}\eta I\left(t\right)\text{d}t}{Q_{\text{rated}}}. \end{array}$$

SOC_0_ indicates the initial charge state of the battery. *η* indicates the charging and discharging efficiency. *Q*_rated_ indicates the rated capacity of the battery. (*t*) indicates the current value at time *T*, which is greater than 0 indicates discharge, and less than 0 indicates charging. The SOC of lithium-ion batteries is between 0 and 1. Under ideal conditions, when the charge runs out, the SOC = 0, and for a fully charged new battery, the SOC = 1.

At present, the SOC estimation methods are as follows from Figure 1.

### 3.2. Fully Connected Neural Network

Fully connected neural networks apply all input parameters to the hidden layer.  Figure 2 shows a three-layer network. In real conditions, the hidden layer [10, 19, and 20] can have many fully connected neural networks.

In this paper, *D* represents the meaning of the scale. Different network layers have different values of D. It shows how many features there are. *x*_1_, *x*_2_,…… *x*_*d*_ mean that there are *d* characteristic inputs. Let *m*_1_, *m*_2_, *m*_3_,…… *m*_*d*_ represent features with *d* hidden layers. Different network layers have different eigenvalues. *h*_1_, *h*_2_……, *h*_*d*_ represent the number of features of the second hidden layer. *o*_1_ represents the value of the output of the multilayer perceptron network. W represents the weight of each feature. B is the offset. Capital W and *X* and *M* are matrices. *f*(·) represents the activation function. This function generally has a nonlinear function.

(3) $$\begin{array}{c} z=\left(\sum_{d=1}^{D}w_{d}^{1}x_{d}\right)+b=W_{1}^{T}X+b,\\ m=f\left(z\right),\\ s=\left(\sum_{d=1}^{D}w_{d}^{2}m_{d}\right)+b=W_{1}^{T}M+b,\\ h=f\left(s\right),\\ o=\left(\sum_{d=1}^{D}w_{d}^{3}h_{d}\right)+b. \end{array}$$

We usually express *f* of *x* as the activation function. There are many options for activation functions. The following functions are commonly used.

(4) fx=σx=Sigmoidx=11+e−x,fx=tanhx=ex−e−xex+e−x,fx=ReLUx=MAX0,x,fx=Mishx=x∗tanh1+ex.

Different activation functions are used to train the network in the same network layer.

This paper mainly belongs to the regression model. So the loss function uses the mean square error loss function. *Y*_*n*_ represents the actual value, while *O*_*n*_(*x*) represents the value predicted by the model after multilayer neural network training [20].

(5) $$\begin{array}{c} J\left(w\right)=L\left(x,y,w\right)=MSE=\frac{1}{N}\sum_{n=1}^{N}{\left(Y_{n}-O_{n}\left(x\right)\right)}^{2},\\ J\left(w\right)=L\left(x,y,w\right)=RMSE=\sqrt{\frac{1}{N}\sum_{n=1}^{N}{\left(Y_{n}-O_{n}\left(x\right)\right)}^{2}}. \end{array}$$

The parameter updating optimization includes the stochastic gradient descent method and the Adam optimization method [21]. The calculation steps of stochastic gradient descent are as follows:

(6) $$\begin{array}{c} \nabla_{w}J\left(w\right)=\frac{1}{N}\sum_{n=1}^{N}\nabla_{w}L\left(x^{n},y^{n},w\right),\\ w=w+\alpha *\nabla_{w}J\left(w\right). \end{array}$$

Ideally, the gradient should be updated after all the training samples have been calculated. However, in practical conditions, due to computer computing power and time consumption, the small-batch stochastic gradient descent method is generally used for gradient updating. K means training samples in small-batch. The random gradient descent method in the small-batch is adopted. K is less than N. *α* is the learning rate, which determines the speed of gradient advance.

(7) $$\begin{array}{c} g=\frac{1}{K}\nabla_{w}\sum_{k=1}^{K}L\left(x^{k},y^{k},w\right),\\ w=w+\alpha *g. \end{array}$$

The small-batch stochastic gradient descent method [22] has a slow convergence rate. Therefore, the Adam gradient update algorithm can be used. Adam algorithm has the advantages of very efficient calculation and less memory. Adam algorithm has the following hyperparameters *β*_1_, *β*_2_ and *ε*. The update from time *t* to time *t*+1 is as follows:

(8) $$\begin{array}{c} g_{t+1}=\nabla_{w}J\left(w_{t}\right),\\ v_{t+1}=\beta_{1}*v_{t}+\left(1-\beta_{1}\right)*g_{t},\\ s_{t+1}=\beta_{2}*s_{t}+\left(1-\beta_{2}\right)*g_{t}^{2},\\ {\bar{v}}_{t+1}=\frac{v_{t+1}}{\left(1-\beta_{1}^{t}\right)},\\ {\bar{s}}_{t+1}=\frac{s_{t+1}}{\left(1-\beta_{2}^{t}\right)},\\ w_{t+1}=w_{t}-\alpha *\frac{{\bar{v}}_{t+1}}{\left(\sqrt{{\bar{s}}_{t+1}}+\varepsilon \right)}. \end{array}$$

In actual training, the most important is to standardize the data. *X*_min_ represents the minimum value of the feature column. *X*_max_ represents the maximum value of the feature column.

(9) $$\begin{array}{c} X=X*\frac{X-X_{\min}}{X_{\max}-X_{\min}}. \end{array}$$

### 3.3. Improved Multilayer Perceptron Algorithm

However, the simple and shallow multilayer perceptron algorithm is insufficient to meet the requirements. The multilayer perceptron algorithm also needs to change. First, the BatchNormalization layer has been added for input to the fully connected network. BN means BatchNormalization layer. The BatchNormalization layer can improve the stability of network training depth. Second, the width of the fully connected neural network is changed. The width of the fully connected network is also a key factor affecting the algorithm's accuracy. Its value range is [30, M]. *M* is a positive integer greater than or equal to 30. Third, the activation function changes. By changing the activation function to adapt to the lithium-ion battery data, the most suitable activation function for lithium-ion battery data was found. Fourth, in order to prevent over-fitting of the depth multilayer perceptron algorithm, the Dropout layer is added to perform pruning. Finally, to increase the network depth of multilayer perceptrons, a BatchNormalization layer plus a fully connected neural network plus an activation function layer plus a Dropout layer is defined as a Block in this paper. The depth of the whole algorithm model can be increased by increasing the depth of the Block layers. The value of the Block layer is [3, N]. The value of N is a positive integer greater than 3. FCN stands for the fully connected neural network.

The activation function selection range is Sigmoid and tanh and ReLU and Mish. The width *M* of FCN(fully connected neural network) is roughly 30 and 50 and 80 and 150 and 300. The most suitable FCN width for a lithium-ion battery was selected by testing. The value of Block Number ranges from 3 to 11. The network depth with better performance is chosen as the final network depth of the algorithm.  Figure 3 shows the improved multilayer perceptron algorithm.

## 4. Experiments

This article uses an open dataset. The battery test data came from the Centre for Advanced Life Cycle Engineering (CALCE) Battery Research Group of the University of Maryland. The battery models and detailed information used in this document are shown in Table 1.

Since the estimation process of SOC is a continuous process, the SOC value at *t* time has great reference significance to the SOC value at *t* +  1 time. Therefore, this paper preprocessed the training data. Discard the data in the first line and take the SOC value of the data in the first line as a characteristic parameter of the data in the second line, recursively in turn. In addition, because the values of InternalResistance, IsFCData, ACImpedance, and ACIPhaseAngle have not changed, the estimation relationship between these four characteristic values and SOC is zero after thermal analysis. Therefore, in this paper's training and testing process, these four features were removed, and the feature UPValue was added. In addition, in the pretreatment process, some standardized processing is done for these features, which is more conducive to the convergence of the model algorithm.

The battery parameters and initial capacity tested in the dataset are shown below in Figure 4.

Initial capacity testing is critical to determine the accurate SOC of lithium batteries. It determines the value of the initial SOC when the SOC is first evaluated. But the initial capacity itself is also temperature-dependent. Therefore, when testing the initial capacity, it is necessary to add the characteristic parameter of temperature to determine the initial capacity. In this paper, the lithium-ion battery is mainly tested at 25 degrees Celsius, so it needs to test its initial capacity at 25 degrees Celsius. Initial capacity testing can be done in two general ways. The first is LowCurrent OCV. It used C/20 or C/25 to charge and discharge the battery so that the corresponding terminal voltage is an approximation of Incremental Current OCV.

The actual running process of the electric vehicle is quite complicated. To simulate the engineering reality of these electric cars, there are generally FUDS(The Federal Urban Driving Schedule), DST(Dynamic Stress Test), US06(Urban Dynamometer Driving) Schedule, and BJDST(Beijing Dynamic Stress Test). In this paper, FUDS and BJDST [3, 23–26] are used to test procedures through these two working conditions to test the multi-neural network training test.

The test results are as follows in Figure 5 when the temperature is 25 degrees Celsius under FUDS condition.

The test results are as follows in Figure 6 when the temperature is 25 degrees Celsius under the BJDST condition.

In general, PCA [27] is performed on the columns of the dataset. This removes columns that are not closely related to the target column. PCA operation can improve the speed of matrix operation. However, there are fewer columns in this dataset. In this case, PCA is a waste of time.  Figure 7 is a thermal diagram of column relationships.

## 5. Result and Discussion

In the design of a multilayer perceptron algorithm, different network depths are used to evaluate the error of SOC estimation. Through the design of different network depths, relatively good network depth is selected as the standard network model for SOC estimation. This paper involves a total of three-layer neural networks to eleven-layer neural networks. The network depth which is most suitable for SOC estimation of lithium-ion batteries is examined by different network depths. This article uses 30% of the dataset as the testing dataset. 70% of the dataset is the training dataset. The number of training cycles is initialized to 50. Epoch = 50. Select 64 for small batch quantity and BatchNum = 64. The hyperparameter of the learning rate was set at 0.001. The data set was divided into BJDST and FUDS, which performed differently for different network depths. In this paper, the depth of the network is tested separately. Figures 8 and 9 show the training errors tested at different network depths.

In the FUDS test, the training network uses a total of three-layer to ten-layer neural networks, and it can be seen that nine-layer neural networks and eight-layer neural networks perform better. However, the advantage of network depth has not been shown due to the small gap between network layers and the small number of cycles. Therefore, eight-layer neural networks and ten-layer neural networks were selected as the comparative experimental parameters for different epochs in the future. It is the equivalent of setting up a controlled trial like group A and group B. It can be seen from BJDST that the performance of a six-layer neural network and ten-layer neural network is better. Therefore, in the BJDST data set, this paper chooses the comparison test after a six-layer neural network and a ten-layer neural network. This can test the effect of neural networks with different depths as the epoch increases. The following Figures 10 and 11 show the performance of two groups of neural network depths under the same epochs. At the same time, the performance of training errors of different network depths under different epochs can also be seen.

With the increase in the number of epoch cycles, the training error gradually decreased. In addition, it can be seen from the FUDS data set that when the epoch is greater than 60, the training error of the ten-layer neural network is smaller than that of the eight-layer neural network. It can be seen from the experimental results in this paper that with the increase in the number of epoch, the performance of the deep neural network is better than that of the shallow neural network. In the BJDST data set, the performance gap between a six-layer neural network and a ten-layer neural network is not particularly obvious. But when the epoch equals 100, the training error of a ten-layer neural network is better than that of a six-layer neural network.

Network width is also a key factor affecting the performance of deep learning algorithms. When the width of the network is small, it cannot extract many features, which will affect the expression ability of the deep learning algorithm. However, the wider the network width is not better; too wide a network is prone to an over-fitting phenomenon. The main idea of this paper is this. When comparing network width and network depth, this paper gives priority to increasing network depth rather than network width. This idea is also in line with the idea of the deep learning algorithm.

As shown in Figure 12, the best results are achieved when the network width is 300. However, when the network width increases from 150 to 300, the test error is not significantly reduced. Therefore, the maximum network width selected in this paper is 150.

Table 2 shows the training errors of different activation functions. The data in Table 2 were tested when the neural network width was 150, the network depth was 10, and the epoch was 100.

Under the above conditions, the ReLU activation function has the smallest training error and performs best. Tests for the rest of this article use the ReLU activation function. However, as the network depth increases, there is a high probability that Mish activation functions will outperform ReLU activation functions. This paper is limited to optimal local selection under current conditions.

Ten-layer neural network was used to compare the test errors. A unified neural network model was used to train FUDS and BJDST datasets simultaneously. This can improve the robustness of the design algorithm model. The ten-layer neural network model algorithm designed in this paper is compared with other algorithms when the epoch is equal to 100, and the maximum network width is equal to 150.

The comparison of the test errors of the FUDS test and the BJDST test from different methods is shown in Figures 13 and 14.

This article estimates the SOC of the test dataset on BJDST and FUDS, respectively, as shown in Figures 15 and 16.

SVM refers to support vector machine [7]. LSTM refers to long short-term memory [7, 18, 21]. RNN means recurrent neural network [3, 28]. EKF means extended Kalman filter [29, 30]. ACKF means adaptive cubature Kalman filter. PF refers to particle filter. GSA represents Genetic simulated annealing algorithm [31, 32]. RBFNN represents Radial Basis Function Neural Network [32, 33]. The comparison between the test errors of the FUDS test set and different methods is shown in the following Table 3.

The test errors of the BJDST [32] test set are compared with different methods in the following Table 4.

There are some good methods to reduce errors, such as enhancing datasets and training deeper neural networks, which have not been used. In addition, an attention mechanism can better improve accuracy and reduce training error and test error, which is not used in this paper. Future work will be to use better methods to estimate SOC more accurately.

## 6. Conclusions

The structure of the improved multilayer perceptron algorithm meets the need for SOC estimation of lithium-ion batteries. The convergence and accuracy of the algorithm are accelerated by adding a Dropout layer and a BatchNormalization layer to the full connection layer.

Meanwhile, this article compares the effects of the Sigmoid activation function, tanh activation function, Relu activation function, and Mish activation function on the improved multilayer perceptron algorithm. Relu activation function and Mish activation function are relatively accurate. The depth of the neural network is also a key factor affecting algorithm performance. A block designed in this article is the first layer, which contains the BatchNormalization layer, a fully connected neural network layer, an activation function layer, and a dropout layer. Blocks of three to eleven layers are selected for comparison. Finally, the 10-layer block is selected with relatively good network depth. The width of neural network has a significant influence on the performance of neural networks. This article compares the width of 50, the width of 80, the width of 120, the width of 150, and the width of 300. A maximum width of 150 was selected. It is because maximum widths of 150 and 300 have very little effect on algorithm performance. According to Occam's Razor principle, the maximum width is 150, which can not only reduce the complexity of the algorithm but also reduce the training time, and meet the requirements of SOC estimation for lithium-ion batteries. Finally, relatively suitable network depth and network width are selected to meet the needs of lithium-ion battery SOC estimation.

The algorithm designed during this article also can be applied to many fields. The algorithm during this paper can be applied to the prediction of SOH, SOE, and also the operation of an aero-engine field.

## Figures and Tables

**Figure 1:** SOC estimation methods.

**Figure 2:** Multilayer perceptron network architecture.

**Figure 3:** Improved multilayer perceptron algorithm.

**Figure 4:** Voltage and current curve in the initial capacity test of lithium-ion battery.

**Figure 5:** FUDS test voltage and current at 25 degrees Celsius.

**Figure 6:** BJDST test voltage and current at 25 degrees Celsius.

**Figure 7:** Relational heat maps in datasets.

**Figure 8:** Training errors of different network depths during FUDS testing.

**Figure 9:** Training errors of different network depths during BJDST testing.

**Figure 10:** Training error curves under the different epochs of the FUDS dataset.

**Figure 11:** Training error curves under the different epochs of the BJDST dataset.

**Figure 12:** Training error curves under the different epochs of the BJDST dataset.

**Figure 13:** Test errors of different methods under the FUDS dataset.

**Figure 14:** Test errors of different methods under the BJDST dataset.

**Figure 15:** SOC estimation on FUDS testing dataset.

**Figure 16:** SOC estimation on BJDST testing dataset.

**Table 1:** Details of the batteries used in the experiment.

Type	Detail
Battery cell	INR 18650-20R
Nominal capacity	2000mAh
Cell chemistry	LNMC/Graphite
Upper cut-off voltage	4.2 V
Lower cut-off voltage	2.5 V
Nominal voltage	3.6 V
Dimensions(mm)	18.33 ± 0.07 mm
Usage temperature	0–50°C

**Table 2:** Training errors in different activation functions.

Activation function	DataSet	TrainLoss
Sigmoid	FUDS	5.62
tanh	FUDS	1.37
ReLU	FUDS	0.09
Mish	FUDS	0.35
Sigmoid	BJDST	7.32
tanh	BJDST	2.11
ReLU	BJDST	0.21
Mish	BJDST	0.76

**Table 3:** Test errors of different methods on FUDS dataset.

ID	Methods	RMSE
1	SVM	3.28
2	LSTM	2.49
3	SVM-PF	1.65
4	LSTM-ACKF	2.2
5	RNN	2.73
6	LSTM-PF	1.5
7	RNN-PF	1.25
8	MLP	0.96

**Table 4:** Test errors of different methods on BJDST dataset.

ID	Methods	RMSE
1	EKF	1.95
2	BPNN-GSA	0.95
3	ECM	3.01
4	ELM-GSA	0.76
5	RBFNN-GSA	1.12
6	MLP	0.68

## Data Availability

All data used to support the findings of the study are included within the article.
